The article "Centre of pressure parameters for the assessment of biomechanical risk in fatiguing frequency-dependent lifting activities" was published in 2022. Journal: PLoS One.

# Centre of pressure parameters for the assessment of biomechanical risk in fatiguing frequency-dependent lifting activities

**DOI:** 10.1371/journal.pone.0266731

**Published:** 2022-08-10

**Authors:** Carmen D’Anna, Tiwana Varrecchia, Alberto Ranavolo, Alessandro Marco De Nunzio, Deborah Falla, Francesco Draicchio, Silvia Conforto

**Affiliations:** 1 Department of Engineering, Roma Tre University, Roma, Lazio, Italy; 2 Department of Occupational and Environmental Medicine, Epidemiology and Hygiene, INAIL, Monte Porzio Catone, Rome, Italy; 3 LUNEX International University of Health, Exercise and Sports, Differdange, Luxembourg; 4 Luxembourg Health & Sport Sciences Research Institute A.s.b.l., Differdange, Luxembourg; 5 Centre of Precision Rehabilitation for Spinal Pain (CPR Spine), School of Sport, Exercise and Rehabilitation Sciences, University of Birmingham, Edgbaston, United Kingdom; Duke Kunshan University, CHINA

## Abstract

Lifting tasks, among manual material handling activities, are those mainly associated with low back pain. In recent years, several instrumental-based tools were developed to quantitatively assess the biomechanical risk during lifting activities. In this study, parameters related to balance and extracted from the Centre of Pressure (CoP) data series are studied in fatiguing frequency-dependent lifting activities to: i) explore the possibility of classifying people with LBP and asymptomatic people during the execution of task; ii) examine the assessment of the risk levels associated with repetitive lifting activities, iii) enhance current understanding of postural control strategies during lifting tasks. Data were recorded from 14 asymptomatic participants and 7 participants with low back pain. The participants performed lifting tasks in three different lifting conditions (with increasing lifting frequency and risk levels) and kinetic and surface electromyography (sEMG) data were acquired. Kinetic data were used to calculated the CoP and parameters extracted from the latter show a discriminant capacity for the groups and the risk levels. Furthermore, sEMG parameters show a trend compatible with myoelectric manifestations of muscular fatigue. Correlation results between sEMG and CoP velocity parameters revealed a positive correlation between amplitude sEMG parameters and CoP velocity in both groups and a negative correlation between frequency sEMG parameters and CoP velocity. The current findings suggest that it is possible to quantitatively assess the risk level when monitoring fatiguing lifting tasks by using CoP parameters as well as identify different motor strategies between people with and without LBP.

## 1. Introduction

Work-related low back disorders (WLBDs), covering both low back pain (LBP) and low back injuries, are a common and costly occupational health condition associated with significant work productivity loss and work absenteeism resulting in disability payment [1, 2]. Among manual material handling activities, lifting tasks are those mainly associated with the development of WLBDs [3–5]. Despite improved working conditions facilitated by automation of some tasks, manual material handling remains in many occupational fields (e.g. industry, agriculture, construction sector) [6].

The article "Centre of pressure parameters for the assessment of biomechanical risk in fatiguing frequency-dependent lifting activities" was published in 2022. Journal: PLoS One.

A precise and accurate biomechanical risk assessment is relevant to prevent the onset of WLBDs and to evaluate the effectiveness of ergonomic interventions [4, 7–10]. Among other approaches, the Revised National Institute for Occupational Safety and Health (NIOSH) Lifting Equation (RNLE) [2, 4, 11, 12] is the most widely used approach for the biomechanical risk assessment of lifting heavy loads. However, due to equation and parameter restrictions [13, 14], the RNLE cannot be applied in different working conditions such as lifting while seated or kneeling, in a restricted workspace, unstable objects [2] (an object in which the location to the centre of mass varies significantly during the lifting activity, such as liquid containers or partially filled bags, etc.), while carrying, pushing or pulling and in unfavourable environments (i.e. temperature significantly outside 19–26 degrees Celsius range and relative humidity outside 35–50% range) [2]. Furthermore, approximately 35% of the lifting tasks cannot be assessed as at least one of the parameters of the RNLE (horizontal distance, vertical location and displacement of the load, asymmetry angle, lifting frequency, quality of gripping) is outside the accepted ranges.

In recent years, several instrumental-based assessment tools for biomechanical risk assessment have been designed, developed [15, 16] and optimized by the use of machine-learning techniques [17, 18]. These quantitative approaches rely on the computation of kinematic, kinetic and surface electromyography (sEMG)-based indices [16, 19–21] sensitive to different lifting risk conditions and positively correlated to compressive and shear forces at the sacral-lumbar region of the spine. They have significant advantages as they are applicable in scenarios where RNLE cannot be applied [15, 19]. Furthermore, the computational cost for indices calculation is very low, and the recording of signals from the human body can be achieved with unobtrusive, wireless, wearable, miniaturized and low power consumption sensors (i.e. inertial measurement units (IMUs), wireless shoe insoles for ground reaction force measurement and bipolar sEMG probes) [16, 19].

The article "Centre of pressure parameters for the assessment of biomechanical risk in fatiguing frequency-dependent lifting activities" was published in 2022. Journal: PLoS One.

Some studies have examined postural strategies during lifting and analyzed their effect on balance control [22–24]. In the general framework of human movement analysis, postural strategies are typically studied by quantifying the Centre of Pressure (CoP) since it characterizes the whole-body position and depends on body posture control [23]. It has been demonstrated that an altered posture during lifting tasks could induce back pain [22, 25] and increases the risk of slips, trips and falls [24]. Among variables of interest for postural control analysis, measures extracted from the CoP are helpful to study how balance during lifting can be altered by different weights and lifting postures [24]. In particular, the CoP velocity represents an effective parameter to classify different groups of participants [26] depending on the lifting tasks, given its strong correlation with the acceleration of the Centre of Mass (CoM) [27].

Even if the CoP and its derived parameters have been used to provide insight on different postures adopted during lifting activities [26] and has been used to assess the possible influence of altered balance on the risk of slips, falling, and developing neuromuscular disorders, these parameters have not been examined for their potential as quantitative indicators of biomechanical risk for lifting activities.

In this study, we examine whether i) CoP velocity can be used to classify people with LBP from asymptomatic people during the execution of repetitive lifting activities; ii) CoP velocity can be effective in assessing the risk levels associated with repetitive lifting activities iii) changes in measures of the CoP correlate with changes in established sEMG measures of muscle activity typically used as indicators of muscular fatigue.

## 2. Materials and methods

### 2.1 Participants

Fourteen (9 female and 5 males; age: 27.6±3.85 years; body mass index (BMI): 25.26±3.21 kg/m^2^) young, healthy control participants (HC) and seven (3 female and 4 males; age: 25.17±6.43 years; BMI: 23.21±4.39 kg/m^2^) people with LBP were enrolled. All the participants with LBP reported pain bilaterally.

The following eligibility criteria were applied: both HC and LBP had to have the capacity to give informed written consent. HC should not have a history of back or lower limb pain or injury that limited their function and/or required treatment from a health professional over the last three years. People with LBP needed to present with LBP for at least 3 months with pain on at least half of the days over the past 6 months. People with LBP were excluded if they were diagnosed with a specific form of LBP or had serious spinal pathologies. Exclusion criteria for both groups were concurrent systemic, rheumatic or neuro-musculoskeletal disorders, current pregnancy, currently on high doses of opioids (> 30 mg of morphine equivalent dose). Furthermore, to have a homogeneous sample, LBP participants actively seeking treatment for their LBP by therapists (physiotherapist, osteopath, chiropractor etc) within the last three months from the date of enrollment were excluded.

The article "Centre of pressure parameters for the assessment of biomechanical risk in fatiguing frequency-dependent lifting activities" was published in 2022. Journal: PLoS One.

All participants gave their informed written consent before taking part in the study, which was conducted according to the Declaration of Helsinki at the Centre of Precision Rehabilitation for Spinal Pain (CPR Spine), the University of Birmingham, approved by the School of Sport, Exercise & Rehabilitation Sciences Ethics Committee (protocol number MCR260319-1). No information regarding the expected results were provided to the participants to avoid biasing results.

### 2.2 Experimental procedure

The participants performed lifting tasks in three different lifting conditions selected to obtain Lifting Index (LI) values equal to 1, 2, and 3. LI was calculated as the ratio between the actual weight of the lifted load (L) and the recommended weight limit (RWL). RWL provided an estimate of the level of physical demand associated with the lifting task [2] and was calculated according to the RNLE as:

RWL=LCxHMxVMxDMxAMxFMxCM (1)

where LC is the load constant of 23 kg, HM, VM, DM and AM are the horizontal distance, vertical distance, vertical displacement and asymmetry multipliers. They are dimensionless multipliers ranging from 0 to 1 and calculated from the corresponding parameters of interest (horizontal distance (H), vertical location (V), vertical travel displacement (D) and angle of asymmetry (A), Fig 1) by using equations or tables presented in NIOSH method [2, 11]. CM is the coupling multiplier for the quality of gripping, and FM is the frequency multiplier depending on lifting frequency (F), lifting duration and vertical location [2].

**Fig 1:** Experimental setup and cycles definition. Description of the experimental setup (left). Displacement and velocity of an IMU placed on the load (right). Lifting cycle events as black dots (see 2.4.1 for further details).

To define a fatiguing lifting task [2] with different level of risk we have designed the experimental setup as follows [28]: the F values were set at 4 lift/min (FM = 0.83), 11 lift/min (FM = 0.41) and 15 lift/min (FM = 0.28). The other parameters were set constant across all the risk conditions: L = 10 kg, H = 44 cm (HM = 0.57), V = 75 cm (VM = 0.99), D = 40 cm (DM = 0.93), A = 0° (AM = 1). The hand-to-object coupling (C) was defined as “good” (CM = 1). Therefore, the evaluated RWL values were 10, 5 and 3.33 for LI equal to 1, 2 and 3, respectively.

The article "Centre of pressure parameters for the assessment of biomechanical risk in fatiguing frequency-dependent lifting activities" was published in 2022. Journal: PLoS One.

Standing in a neutral body position [2, 29], the participants were asked to lift a plastic crate (34x29x13 cm) with handles using both hands. The three lifting conditions were tested across three non-consecutive days, one testing session per day. The three lifting conditions were randomly assigned across the three testing days to avoid the confounding factor resulting from a predefined order of the risk condition sequence. Testing sessions were 78 hours apart and at the same time of the day to avoid confounding effects due to fatigue or daily habits. Within each session, the participants performed continuous lifting cycles for 15 minutes. Participants with LBP were asked to perform the lifting cycles to the point of exhaustion if they lasted less than 15 minutes. Specifically, metronome was used to cue the lifting frequency: each time the acoustic signal was heard, the participants raised the load to the defined height (Fig 1), they released it by standing upright and waited for the next acoustic signal.

### 2.3 Data recording

Kinematic (from an IMU sensor), kinetic (from a Wii-Fit Balance Board) and electromyography (from bipolar surface electrodes) data were acquired simultaneously. All the sensors were synchronized with a trigger signal generated by a synching device (MyoSync, Noraxon).

#### 2.3.1 Kinematic recording

An inertial sensor (myoMotion Research PRO IMU, Noraxon) placed on the plastic crate (z-axis in the vertical direction) was used to acquire load movements and define the lifting cycle. The sampling frequency for the inertial sensors was set at 200 Hz.

#### 2.3.2 Kinetic recording

A Nintendo Wii Balance Board (see Fig 2) operated via an open-source code from the University of Colorado’s Neuromechanics Lab (http://spot.colorado.edu/~alaa/neuro_lab/cu_wii.html) was used to record kinetic data (four vertical forces at the four corners of the balance plate) at a sampling frequency of 30 Hz. The force signals were used to calculate the CoP displacements in both medio-lateral (ML) and antero-posterior (AP) directions, as:

$${CoP}_{AP}=\frac{Y}{2}\frac{\left(F_{4}+F_{1})-(F_{3}+F_{2}\right)}{F_{1}+F_{2}+F_{3}+F_{4}}$$ (2)

$${CoP}_{ML}=\frac{Y}{2}\frac{\left(F_{4}+F_{3})-(F_{1}+F_{2}\right)}{F_{1}+F_{2}+F_{3}+F_{4}}$$

where X and Y represent the distance (in mm) between each force transducer positioned in the centre of each foot-peg, and CoP_ML_ and CoP_AP_ represent the CoP displacement (in mm) calculated in the ML and AP directions, respectively [30]. The Balance Board was calibrated before each acquisition [31].

The article "Centre of pressure parameters for the assessment of biomechanical risk in fatiguing frequency-dependent lifting activities" was published in 2022. Journal: PLoS One.

**Fig 2:** Wii balance board: Reference system and vertical forces recorded at the four corners F1, F2, F3, F4. Y-axis and X-axis are associated with antero-posterior and medio-lateral directions, respectively.

#### 2.3.3 Electromyography recording

Muscle activity was acquired (sampling frequency 2000 Hz) via two wireless bipolar sEMG sensors (Ultimium EMG system, Noraxon, USA Inc. Scottsdale, AZ) bilaterally from the erector spinae longissimus (ESL) according to guidelines for electrode placement [32, 33].

### 2.4 Data analysis

Data were processed using Matlab (version 2018b 9.5.0.1178774, MathWorks, Natick, MA, USA) software.

#### 2.4.1 Definition of the lifting and lowering cycles

The vertical displacement and velocity of the IMU placed over the crate were calculated by integrating the filtered acceleration signal (3rd order low-pass Butterworth filtered by applying a 10Hz cut-off frequency) once and twice, respectively. The drift was corrected assuming null vertical speed and acceleration before and after lifting. Each whole-lifting cycle was subdivided into lifting and lowering phases. The onset and termination of the lifting phase were defined as the times the IMU velocity exceeded a threshold of 0.025 m/s along the vertical axis and the maximum point of the vertical displacement of the IMU, respectively [15, 28]. Termination of the lowering phase corresponded to the IMU velocity falling below the 0.025 m/s threshold (see Fig 1) [15]. After the definition of the cycles, a Dynamic Time Warping approach [34] was used to align the curves that were shifted if wrong events were detected [28].

#### 2.4.2 CoP

CoP data were stored for off-line post-processing, which included digital low-pass filtering at a cut-off frequency of 10 Hz. For the whole-lifting cycle task and for both the lifting and lowering phases, twelve parameters were calculated as follows [35]:

- **Spatial parameters:** the range of the CoP in the ML (Range_ML_) and AP (Range_AP_) direction, defined as the difference between the maximum and minimum values of the time series; the mean amplitude (MA) defined as the average distance of the CoP displacement from the mean value; the total lengths of the sway path (SP, SP_ML_ and SP_AP_) defined as the sum of the distances between consecutive points of the 2D CoP path (SP) and along the ML (SP_ML_) and AP (SP_AP_) directions.
- **Frequency domain parameters:** the mean power frequency in both the CoP directions (MPF_ML_ and MPF_AP_,) was extracted from the CoP_AP_ and CoP_ML_ time series density spectrum.
- **Temporal-spatial parameters:** the total mean velocity (MV) of the CoP, and in both ML (MV_ML_) and AP (MV_AP_) directions; the sway area (SA) estimated as the area enclosed by the CoP path per unit of time calculated by summing the area of the triangles formed by two CoP consecutive points and the mean CoP [36].

The article "Centre of pressure parameters for the assessment of biomechanical risk in fatiguing frequency-dependent lifting activities" was published in 2022. Journal: PLoS One.

#### 2.4.3 sEMG parameters

The raw sEMG data of each lifting cycle were band-pass filtered using a fourth-order Butterworth filter of 20–400 Hz to reduce artefacts and high-frequency noise [37, 38]. These signals were analyzed in both time and frequency domains:

- **Time domain:** the root mean square (RMS) within each cycle was calculated on the envelope of sEMG signal obtained with the full-wave rectification and low-pass filtering (fourth-order Butterworth filter at 5 Hz [18, 19, 39]. The envelopes were time-normalized (200 samples using a linear interpolation procedure) to the duration of the whole-lifting cycle [28].
- **Frequency domain:** the mean frequency (MNF) within each whole-lifting cycle was calculated on the power spectral density, estimated using Yule-Walker’s approach: the autoregressive parameters were estimated using Levinson Durbin recursion with a model order p = 15 [19, 40].

For each condition (LI = 1, 2 and 3), the EMG data, related to all the whole-lifting cycles, were amplitude-normalized to the initial value (first cycle of the lifting repetition) [41]. By performing this amplitude-normalization, normalization to a maximum voluntary contraction was not necessary.

### 2.5 Statistical analysis

The statistical analysis was performed using Matlab software (version 2018b 9.5.0.1178774, MathWorks, Natick, MA, USA) to verify the difference between groups, and the effect of the risk levels on CoP parameters considering all lifting repetitions (data were time-averaged in all lifting repetitions), at each minute (data were time-averaged over one-minute windows to compare data with a different number of repetitions of the lifting cycles [28]) for whole-lifting cycle, lifting and lowering phases, separately.

For each CoP parameter, the normality of data distribution was checked using the Shapiro-Walk test. For each group, one-way repeated-measures analysis of variance (ANOVA) or corresponding Friedman t-test (when data was not normally distributed) was performed to determine whether LI levels induce significant changes in each parameter. We reported the F values for ANOVA, Chi values for Friedman test and the degrees of freedom (df) values associated with statistic tests. Post-hoc analyses were performed using a paired t-test with Bonferroni corrections when significant differences were observed. Furthermore, for each LI, the unpaired two-sample t test or Mann-Whitney (MW) test was used to evaluate differences in CoP parameters between groups.

The article "Centre of pressure parameters for the assessment of biomechanical risk in fatiguing frequency-dependent lifting activities" was published in 2022. Journal: PLoS One.

Additionally, to study the statistical difference between the start and the end of the entire task duration, for both groups, the one-way ANOVA was performed considering the time (first and last minute) as a factor for each LI level.

Finally, for both groups, a correlation analysis was performed using Pearson’s rank correlation coefficient between CoP parameters and EMG parameters, considering the mean values among all the participants across the one-minute windows.

For all the statistical analyses the significance level was set at <0.05 the p-value (probability of obtaining results at least as extreme as the observed results of a statistical hypothesis test, assuming that the null hypothesis is correct).

## 3. Results

### 3.1 COP parameters

#### 3.1.1. Results time-averaged across lifting repetitions

Fig 3 shows the means and standard deviations of all CoP parameters calculated for all repetitions within the lifting phase, the lowering phase and the whole-lifting cycle for each risk condition and in both groups.

**Fig 3:** Centre of Pressure parameters. Mean ± SD for each risk level in both groups for all the Centre of pressure (CoP) parameters considering all repetitions within the entire session, in lifting (A), lowering (B) and whole-lifting (C) phases. HC: healthy control participants; LBP: people with Low Back Pain; Range_AP_ and Range_ML_: range of the CoP in the medio-lateral (ML) and antero-posterior (AP) direction; MA: the mean amplitude; SP: total length of the sway path; SP_ML_ and SP_AP_: total excursion in ML and AP directions; MPF_ML_ and MPF_AP_ mean power frequency in ML and AP directions; MV, MV_ML_ and MV_AP_: mean velocity in the average of the CoP, ML and AP directions; SA: sway area. LI: Lifting index. *Statistical significance (p<0.05).

For the HC (Fig 3, left section in each graph), the average values of all the postural parameters increase as the level of risk increases, in each lifting and lowering phases and in the whole-lifting cycle. In the lifting phase (Fig 3A), LI levels determine significant changes for: Range_AP_, MA, SP, SP_ML_, SP_AP_, MPF_ML_, MPF_AP_, MV, MV_ML_, MV_AP_ and SA (Table 1); while no significant changes were found for Range_ML_ (Table 1). Particularly, the post-hoc analysis showed a significant difference between LI = 1 and LI = 3 for all parameters except Range_ML_. In addition, a significant difference between LI = 2 and LI = 3 was observed for velocity (MV, MV_ML_ and SA) and frequency (MPF_ML_ and MPF_AP_) parameters.

**Table 1:** Statistical analysis effect of the risk levels on CoP parameters.

Parameters	phase	HC	LBP
**Range**_**ML**_ **[mm] **	Lifting phase	F = 1.45, df = 2, p = 0.255	F = 0.4, df = 2, p = 0.679
	Lowering phase	F = 1.16, df = 2, p = 0.329	F = 0.45, df = 2, p = 0.649
	Whole-lifting cycle	F = 1.29, df = 2, p = 0.295	F = 1.03, df = 2, p = 0.387
**Range**_**AP**_ **[mm] **	Lifting phase	F = 4.04, df = 2, p = **0.031**	Chi:5.43, df = 2, p = 0.06
	Lowering phase	Chi:7.38, df = 2, p = **0.023**	Chi:3.71, df = 2, p = 0.156
	Whole-lifting cycle	F:1.05, df = 2, p = 0.366	F:1.38, df = 2, p = 0.289
**MA [mm] **	Lifting phase	F = 6.38, df = 2, p = **0.006**	Chi = 6, df = 2, p = 0.051
	Lowering phase	Chi = 6.86, df = 2, p = **0.032**	F = 2.48, df = 2, p = **0.013**
	Whole-lifting cycle	F = 6.13, df = 2, p = **0.007**	F = 2.76, df = 2, p = 0.103
**SP [mm] **	Lifting phase	F = 4.98, df = 2, p = **0.015**	Chi = 2, df = 2, p = 0.368
	Lowering phase	F = 0.97, df = 2, p = 0.393	F = 0.96, df = 2, p = 0.411
	Whole-lifting cycle	F = 7.13, df = 2, p = **0.003**	Chi = 0.86, df = 2, p = 0.651
**SP**_**ML**_ **[mm] **	Lifting phase	F = 3.46, df = 2, p = **0.046**	F = 0.25, df = 2, p = 0.779
	Lowering phase	F = 1.2, df = 2, p = 0.318	F = 0.22, df = 2, p = 0.806
	Whole-lifting cycle	F = 2.8, df = 2, p = 0.080	F = 0.28, df = 2, p = 0.762
**SP**_**AP**_ **[mm] **	Lifting phase	F = 4.86, df = 2, p = **0.016**	Chi = 2, df = 2, p = 0.348
	Lowering phase	Chi = 6.86, df = 2, p = **0.032**	F = 1.35, df = 2, p = 0.296
	Whole-lifting cycle	Chi = 7, df = 2, p = **0.03**	Chi = 0.86, df = 2, p = 0.651
**MPF**_**ML**_ **[Hz] **	Lifting phase	Chi = 16, df = 2, p<**0.001**	F = 11.04, df = 2, p = **0.002**
	Lowering phase	F = 14.66, df = 2, p<**0.001**	F = 7.83, df = 2, p = **0.007**
	Whole-lifting cycle	Chi = 3, df = 2, p = 0.223	Chi = 10.57, df = 2, p = **0.005**
**MPF**_**AP**_ **[Hz] **	Lifting phase	F = 6.55, df = 2, p = **0.005**	F = 3.71, df = 2, p = 0.056
	Lowering phase	F = 13.74, df = 2, p<**0.001**	F = 6.92, df = 2, p = **0.01**
	Whole-lifting cycle	Chi = 0.57, df = 2, p = 0.752	F = 0.002, df = 2, p = 0.975
**MV [mm/s] **	Lifting phase	F = 10.81, df = 2, p<**0.001**	Chi = 3.71, df = 2, p = 0.156
	Lowering phase	F = 8.08, df = 2, p = **0.002**	F = 8.33, df = 2, p = **0.005**
	Whole-lifting cycle	Chi = 17.29, df = 2, p<**0.001**	Chi = 7.71, df = 2, p = **0.02**
**MV**_**ML**_ **[mm/s] **	Lifting phase	F = 9.94, df = 2, p<**0.001**	Chi = 2.57, df = 2, p = 0.277
	Lowering phase	F = 6.99, df = 2, p = **0.004**	Chi = 6, df = 2, p = **0.049**
	Whole-lifting cycle	F = 9.95, df = 2, p<**0.001**	Chi = 5.62, df = 2, p = **0.049**
**MV**_**AP**_ **[mm/s] **	Lifting phase	F = 10.01, df = 2, p<**0.001**	Chi = 3.43, df = 2, p = 0.180
	Lowering phase	Chi = 13.86, df = 2, p = **0.001**	F = 8.66, df = 2, p **= 0.005**
	Whole-lifting cycle	Chi = 17.71, df = 2, p<**0.001**	F = 6.65, df = 2, p = **0.012**
**SA [mm** ^**2**^ **/s] **	Lifting phase	Chi = 10.43, df = 2, p = **0.005**	Chi = 3.71, df = 2, p = 0.156
	Lowering phase	F = 5.38, df = 2, p = **0.011**	F = 4.01, df = 2, p = **0.046**
	Whole-lifting cycle	Chi = 10.43, df = 2, p<**0.005**	Chi = 3.71, df = 2, p = 0.156

Statistical analysis results of the effect of the risk levels on each Centre of Pressure (CoP) parameters in both groups, considering all lifting repetitions (data were time-averaged in all lifting repetitions) for lifting, lowering and whole-lifting phases. HC: healthy control; LBP: people with Low Back Pain; Range_AP_ and Range_ML_: range of the CoP in the medio-lateral (ML) and antero-posterior (AP) direction; MA: the mean amplitude; SP: total length of the sway path; SP_ML_ and SP_AP_: total excursion in ML and AP directions; MPF_ML_ and MPF_AP_ mean power frequency in ML and AP directions; MV, MV_ML_ and MV_AP_: mean velocity in the average of the CoP, ML and AP directions; SA: sway area. LI: Lifting index. Bold: statistical significance (p<0.05).

The article "Centre of pressure parameters for the assessment of biomechanical risk in fatiguing frequency-dependent lifting activities" was published in 2022. Journal: PLoS One.

Within the lowering phase (Fig 3B), LI levels determine significant changes for: Range_AP_, MA, SP_AP_, MPF_ML_, MPF_AP_, MV, MV_ML_, MV_AP_ and SA (Table 1); while no significant changes were found for Range_ML_, SP and SP_ML_ (Table 1).The post-hoc analysis showed a significant difference for the velocity parameters between the LI = 1 and LI = 3 and for MPF_ML_ between each pair of LI and for MPF_AP_ between LI = 1 and both LI = 2 and LI = 3.

For those with LBP (Fig 3, right section in each graph), no significant effects of LI were observed for all the parameters (Table 1) during the lifting phase (Fig 3A) except for MPF_ML_ (Table 1) where the post-hoc analysis showed a significant difference between LI = 1 and LI = 3.

In the lowering phase of the task (Fig 3B), LI levels determine significant changes for MA, MPF_ML_, MPF_AP_, MV, MV_ML_, MV_AP_ and SA (Table 1); while no significant changes were found for: Range_ML,_ Range_AP_, SP, SP_ML_ and SP_AP_ (Table 1).

The post-hoc analysis showed significant differences between LI = 1 and LI = 3 for all of the velocity (MV, MV_ML_, MV_AP_ and SA) and frequency (MPF_ML_ and MPF_AP_) parameters. Furthermore, a significant difference was observed for MPF_ML_ between LI = 1 and LI = 2.

When comparing data between groups, no significant differences (p>0.05) were found during the lifting phase (see Fig 3A) except for MPF_ML_ where a significant difference (p<0.05) was found for LI = 1. During the lowering phase (see Fig 3B), significant differences (p<0.05) were found in MV for LI = 2 and LI = 3, MV_ML_ for LI = 1, LI = 2 and LI = 3, in MV_AP_ for LI = 2, in MPF_ML_ for LI = 1 and LI = 3 and MPF_AP_ for LI = 3. During the whole-lifting cycle (see Fig 3C) significant differences (p<0.05) were found in MV for LI = 3, MV_ML_ for LI = 1 and LI = 3 and MPF_ML_ for LI = 1.

The article "Centre of pressure parameters for the assessment of biomechanical risk in fatiguing frequency-dependent lifting activities" was published in 2022. Journal: PLoS One.

The analysis of the whole-lifting cycle for HC highlighted that LI levels determine significant changes for MA, SP, SP_AP_, MV, MV_ML_, and SA (Table 1); while no significant changes were found for: Range_ML_, Range_AP_, SP_ML_, MPF_ML_ and MPF_AP_ (Table 1).

The analysis of the whole-lifting cycle for LBP highlighted that LI levels determine significant changes for MPF_ML_, MV, MV_ML_ and MV_AP_ (Table 1); while no significant changes were found for: Range_ML_, Range_AP_, MA, SP, SP_ML_, SP_AP_, MPF_AP_ and SA (Table 1).

Notably, all the velocity CoP parameters are sensitive to the risk level and that the values of MV, MV_ML_ and MV_AP_ calculated for LI = 1 and LI = 3 were significantly different for both groups. Thus, from hereon in, further analysis of MV, MV_AP_ and MV_ML_ will only be reported.

#### 3.1.2. Results time-averaged over one-minute windows

Results of minute by minute extracted parameters across the entire task, are shown in Fig 4. For the HC group, the values of MV and MV_AP_ for all the three risk levels were significantly different starting from the eleventh minute of the task (Fig 4A); the values of MV_ML_ for LI = 1 and LI = 3 were significantly different starting from the second minute of the task (Fig 4A).

**Fig 4:** Centre of Pressure parameters across the 15 minutes lifting. Mean ± SD for each risk level in both groups (healthy control (A) and people with Low Back Pain (B)) for mean velocity in the average of the COP (MV) and in medio-lateral (MV_ML_) and antero-posterior (MV_AP_) directions considering all repetitions within each minute of the entire trail of lifting cycles. LI: Lifting index. *Statistical significance (p<0.05).

In LBP, the values of MV, MV_AP_, MV_ML_ for LI = 1 and LI = 3 risk levels were significantly different starting from the fourth minute of the task (Fig 4B). In HC, the regression line, (Fig 5) estimated for each level of risk, showed an increasing trend for all velocity parameters at LI = 2 and LI = 3, and leading to a significant difference between the start and the end of the tasks (Table 2); in contrast, in LBP the MV_ML_ increased significantly for all three levels of risk.

**Fig 5:** Regression line of the centre of pressure parameters. The regression line for each risk level in both groups (Healthy Control—HC left column and people with Low Back Pain–LBP right column) for mean velocity in the average of the CoP (MV) and in medio-lateral (MV_ML_) and antero-posterior (MV_AP_) directions considering the mean of all repetitions within each minute of entire trail of lifting cycles. LI: Lifting index. *Statistical significance (p<0.05).

The article "Centre of pressure parameters for the assessment of biomechanical risk in fatiguing frequency-dependent lifting activities" was published in 2022. Journal: PLoS One.

**Table 2:** Statistical analysis between the first and last minute of lifting.

	LI	MV [mm/s]	MV_ML_ [mm/s]	MV_AP_ [mm/s]
HC	1	0.784	0.416	0.986
	2	**0.009**	**0.015**	**0.049**
	3	**<0.001**	**<0.001**	**0.001**
LBP	1	0.177	**0.034**	0.278
	2	0.059	**0.016**	0.234
	3	**0.031**	**0.016**	**0.040**

For each risk level in both groups for all the Centre of Pressure (CoP) parameters, the statistical analysis compares the first and last minute considering whole-lifting cycles. HC: healthy control; LBP: people with Low Back Pain; Range_AP_ and Range_ML;_ MV, MV_ML_ and MV_AP_: mean velocity in the average of the CoP, ML and AP directions; SA: sway area. LI: Lifting index. Bold: statistical significance (p<0.05).

### 3.2 sEMG parameters

Fig 6 presents the RMS and MNF mean values and the regression lines for each risk level in both groups.

**Fig 6:** Mean value and regression line of sEMG parameters. Mean value of the root mean square (RMS) and mean frequency (MNF) considering the mean of all the repetitions within each minute of the whole-lifting cycle and the regression line for each risk level in both groups (healthy control (A) and people with Low Back Pain (B)). Each point on the graphs represents the group average extracted every minute.

### 3.3 Correlation between CoP and sEMG parameters

The correlation between sEMG parameters (RMS and MNF) and velocity CoP parameters (MV, MV_ML_ and MV_AP_) are reported in Table 3. Positive significant correlations were found between RMS and MV, MV_ML_ and MV_AP_ at LI = 3 for both groups and between RMS and MV_ML_ at LI = 2 for LBP; significant negative correlations were observed between MNF and MV, MV_ML_ and MV_AP_ at LI = 2 and LI = 3.

**Table 3:** Correlation between CoP and EMG parameters.

		MV -RMS		MV_ML_ -RMS		MV_AP_ -RMS		MV -MNF		MV_ML_ -MNF		MV_AP_ -MNF	
	LI	r	p	r	p	r	p	r	p	r	p	r	p
HC	1	-0.317	0.25	0.003	0.992	-0.378	0.165	0.155	0.58	-0.073	0.796	0.188	0.503
	2	0.245	0.379	0.413	0.126	0.07	0.803	**-0.692**	**0.004**	**-0.709**	**0.003**	**-0.539**	**0.038**
	3	**0.903**	**<0.001**	**0.859**	**<0.001**	**0.894**	**<0.001**	**-0.917**	**<0.001**	**-0.901**	**<0.001**	**-0.895**	**<0.001**
LBP	1	-0.31	0.261	-0.522	0.046	-0.199	0.476	0.215	0.442	0.016	0.955	0.253	0.364
	2	0.408	0.131	**0.638**	**0.011**	0.192	0.493	**-0.7**	**0.004**	**-0.56**	**0.03**	**-0.621**	**0.013**
	3	**0.803**	**<0.001**	**0.848**	**<0.001**	**0.704**	**0.003**	**-0.801**	**<0.001**	**-0.692**	**0.004**	**-0.782**	**0.001**

The r and p values of correlation analysis between the Centre of Pressure (CoP) parameters and EMG parameters for both groups. RMS: root mean square of erector spinae muscle; MNF: mean frequency of erector spinae muscle; MV, MV_ML_ and MV_AP_: mean velocity in the average of the COP, ML and AP directions; HC: healthy control; LBP: people with Low Back Pain. Bold: statistical significance (p<0.05)

The results obtained are summarized in the 3D graph in Fig 7, where the CoP velocity parameters are reported with the EMG amplitude and frequency parameters showing discrimination among the risk levels and supported by the statistical analysis.

The article "Centre of pressure parameters for the assessment of biomechanical risk in fatiguing frequency-dependent lifting activities" was published in 2022. Journal: PLoS One.

**Fig 7:** Relation between CoP and EMG parameters. 3D plot of the Centre of Pressure (CoP) parameters and EMG parameters for both HC and LBP groups. Each point represents the group average extracted every minute (across the 15 minutes lifting). RMS: root mean square of the erector spinae muscle; MNF: mean frequency of the erector spinae muscle; MV, MV_ML_ and MV_AP_: mean velocity for the 2D CoP motion and along the ML and AP directions; HC: healthy control; LBP: people with Low Back Pain.

## 4. Discussion and conclusion

This study demonstrated the possibility to use measures of postural control, and CoP velocity in particular, to classify people with and without LBP during the execution of repetitive lifting activities and also to discriminate the levels of risk associated with those activities as designed by the RNLE. The results also showed that measures of CoP velocity correlate with myoelectric manifestations of muscular fatigue.

The results obtained in the present study highlight that different postural control strategies were adopted by the two groups (i.e. HC and LBP) during the lifting tasks. In particular, during the lifting phase of the task, the asymptomatic group increased the postural oscillations when moving from LI = 1 to LI = 3 as reflected by the increase in postural parameters. The same did not occur for the group with LBP, which adopted a similar postural strategy for the three levels of risk. In the lowering phase of the task, the spatial-time (i.e. velocity of CoP) and the frequency parameters were different between groups and between LI = 1 and LI = 3, in both the antero-posterior and medio-lateral direction (Fig 4). Collectively, these results indicate that, on average, people with LBP adopt different postural strategies during both the lifting and lowering phases, in a repetitive lifting task, compared to asymptomatic people.

The discriminant capacity of CoP parameters, when considering the differentiation between groups and between risk levels, was best examined via the minute by minute analysis (Fig 4). Such an approach demonstrated discriminative power, across the risk levels, for asymptomatic people from the beginning of the task. In contrast those with LBP used the same lifting strategy for the first three minutes, across the risk levels, showing differences from the 4th minute on. Besides a linear increase of the CoP velocity parameters (Fig 5) for both groups, analysis of the EMG parameters also demonstrated a progressive increase of the RMS and decrease of the MNF decrease (Fig 6), consistent with progressive muscle fatigue [42, 43]. Moreover, a significant correlation–at LI = 3 for both groups and at LI = 2 for LBP–between EMG parameters and CoP velocity suggest that the different postural strategy adopted by people with LBP relates to the extent of muscle fatigue experienced during the execution of the task at increasing risk levels [44].

The article "Centre of pressure parameters for the assessment of biomechanical risk in fatiguing frequency-dependent lifting activities" was published in 2022. Journal: PLoS One.

Despite the small sample size and the absence of a gender-based analysis, which could be relevant when examining postural modifications during the execution of a lifting task [26], our findings suggest that it is possible to quantitatively assess the risk level when monitoring fatiguing lifting tasks by using CoP parameters. They extend the possibilities offered by the currently available instrumental-based tools for biomechanical risk classification, which due to their low cost and ease of use, would allow continuous monitoring in different working environments.

In addition, the effectiveness of all the technological solutions mentioned can be improved by the support of real-time biofeedback systems for the self-control of the balance [45], that have been shown to help the correct execution of the task and then to reduce the risk of slips, trips and falls [24].

## Supporting information

S1 File (RAR)
